# Leisure-time physical activity and the risk of metabolic syndrome: meta-analysis

**DOI:** 10.1186/2047-783X-19-22

**Published:** 2014-04-23

**Authors:** Yijun Huang, Xuemei Liu

**Affiliations:** 1 College of Physical Education, Ludong University, Hongqi Middle Road 186, Zhifu District, Yantai 264025, Shandong, China; 2 Reproductive Medicine Center, Yantai Yuhuangding Hospital, Yantai 264000, Shandong, China

**Keywords:** Metabolic disorder, Quantitative review, Blood pressure, Insulin resistance, Glucose intolerance, Sensitivity analysis

## Abstract

**Background:**

The purpose of this study was to assess the association between leisure-time physical activity (LPA) and the risk of metabolic syndrome (MS).

**Methods:**

Prospective cohort studies of the association between LPA and the risk of MS were retrieved from the PubMed and Embase databases up to 12 August 2013. The statistical analysis in this study was performed using Stata 11.0 software. Odds ratios (ORs) and 95% confidence intervals (CIs) were used to evaluate the effect of LPA on the risk of MS.

**Results:**

A total of five articles were included in this meta-analysis. The overall effect sizes indicated that people with moderate level LPA (OR = 0.89, 95% CI: 0.82 to 0.96, *P* = 0.003) or high level LPA (OR = 0.58, 95% CI: 0.38 to 0.89, *P* = 0.012) had lower risk of MS than people with low level LPA. The subgroup analysis by gender showed that high level LPA could reduce the risk of MS in populations of different genders (female, OR = 0.20, 95% CI: 0.08 to 0.49, *P* <0.001; male, OR = 0.59, 95% CI: 0.43 to 0.82, *P* = 0.002). However, compared with low level LPA, Americans with high level LPA did not significantly reduce the risk of MS (OR = 0.59, 95% CI: 0.43 to 0.82, *P* = 0.002), while a significant decrease of the risk of MS was found in Europeans with high level LPA (OR = 0.49, 95% CI 0.32 to 0.77, *P* = 0.002) in the subgroup analysis by region.

**Conclusions:**

The meta-analysis confirmed that a moderate and high level of LPA could reduce the risk of MS.

## Background

Metabolic syndrome (MS) is a common metabolic disorder owing to a combination of unhealthy diet, sedentary lifestyle and genetic predisposition [1]. Studies have shown that it is characterized by the presence of any of the following: abdominal obesity, dyslipidemia, low high-density lipoprotein (HDL), elevated blood pressure, glucose intolerance and insulin resistance [2-4]. As a clustering of risk factors, MS is strongly associated with the incidence of all-cause mortality, endometrial cancer, diabetes and cardiovascular diseases [5-7]. Therefore, it is essential to find appropriate approaches to prevent and control MS-related diseases.

In recent years, the role of physical activity (PA) in health has been increasingly recognized [8]. Generally, PA is defined as any bodily movement produced by skeletal muscles that results in energy expenditure [9]. It is well documented that habitual leisure-time PA (LPA) could play a preventive role in hypertension, insulin resistance, glucose intolerance [10], elevated triglycerides, low level HDL and MS [11]. For MS, Méndez-Hernández and colleagues indicated that at least 30 minutes a day of LPA at different intensity levels significantly reduced the risk of MS among Mexican men and women [12]. However, Cheriyath and co-workers found that LPA was weakly associated with the incidence of MS [13]. In addition, PA during leisure recorded in middle age prior to the current waves of obesity and diabetes had an independent predictive association with the presence of MS [14]. It is clearly observed that inconsistent results exist in the current studies of the association between LPA and MS. This may be the result from the use of different definitions and the characteristics of the included populations. To provide reliable and strong evidence, we conducted a meta-analysis of prospective cohort studies with the aim to assess the association of LPA with the risk of MS.

## Methods

### Search strategy

We performed pre-established search strategies and retrieved literature in a systematic way from the PubMed and Embase databases with a retrieval deadline of 12 August 2013. The keywords used for searching included three aspects: 1) exposure factors (‘physical activity’ , ‘leisure-time physical activity’ , ‘occupational physical activity’ and ‘sport’); 2) MS (‘metabolic syndrome’ , ‘MetS’ , ‘MS’ , ‘metabolic syndrome X’ , ‘syndrome X’ , ‘cardio metabolic risk factor’ and ‘insulin resistance syndrome’); and 3) study type (‘prospective’ , ‘cohort’ and ‘follow up’). In addition, a manual search of paper literature from relevant original studies, the screening of references and the included studies from the related reviews were performed to obtain additional studies.

### Inclusion and exclusion criteria

The studies included in the present meta-analysis met the following criteria: 1) the studies were prospective cohort studies; 2) the study subjects were healthy; 3) the study was designed to assess the effect of PA on the risk of MS; 4) the control group comprised individuals with a low level of PA; and 5) the available data should be provided or calculated out from the data of the studies. The studies were excluded if: 1) the language of the studies was not English; and 2) articles were reviews, letters and comments. In addition, for repeatedly published literature, the studies with the most complete data were included in this meta-analysis.

### Data abstraction and quality evaluation

Two evaluators independently selected studies and extracted data. Discrepancies were resolved by discussion with each other. From the studies that met the inclusion criteria, the following data were abstracted: the first author’s name, year of publication, region, year of the study, duration of follow-up, ascertainment of LPA level, diagnostic criteria of MA, age and gender of the subjects, sample size in each group and the data of statistical analysis.

The quality of the included studies was evaluated according to the Newcastle-Ottawa Scale [15]. This scoring system for cohort studies comprised eight scoring items: representativeness of the exposed cohort, selection of the unexposed cohort, ascertainment of exposure, outcome of interest not present at start of study, control for important factor or additional factor, outcome assessment, follow-up long enough for outcomes to occur and adequacy of follow-up of cohorts. The score of each item was 1, except for the item of control for important factor or additional factor, which was 2. Thus, the total score was nine. The studies with a score of more than 7 were considered high quality studies.

### Statistical analysis

The statistical analysis in this study was performed using Stata 11.0 software (StataCorp LP, College Station, TX, USA). The odds ratio (OR) as well as the corresponding 95% confidence intervals (CIs) in each study were pooled to assess the association between LPA and the risk of MS [16]. Heterogeneity among studies was evaluated by Cochran’s Q test and the *I*^2^ parameter [17]. *P* <0.05 and *I*^2^ > 50% were considered to be heterogeneous. When significant heterogeneity was detected in the studies, the random effects model was used to pool the data. Otherwise, the fixed effects model was used. The subgroup analysis was conducted by gender (male/female) and region (Europe/the Americas) to investigate the influence of these confounding factors on the outcomes of this meta-analysis.

A sensitivity analysis was performed to detect stability and credibility of the outcomes by changing the effects model and the trim-and-fill method [18]. Publication bias was assessed by the funnel plot with Begg’s and Egger’s tests [19,20]. *P* <0.05 was considered statistically significant.

## Results

### Literature retrieval

According to the initial search strategy, we achieved 838 and 550 articles from the Embase and PubMed libraries, respectively. First, a total of 227 repeated and 1,131 obviously irrelevant articles were excluded. Among the remaining 30 studies, we reviewed the titles, abstracts and the full texts. Finally, five articles met the screening criteria and were included in this meta-analysis [12-14,21,22]. There were no additional articles obtained from the manual search (Figure 1).

**Figure 1:** **Literature search and study selection.** CI, confidence interval; OR, odds ratio; PA, physical activity.

### Study characteristics and quality assessment

The characteristics of the included studies are shown in Table 1. Among the five included studies, the subjects in the studies of Méndez-Hernández *et al*. [12] and Yang *et al*. [21] consisted of male and female populations. Thus, a total of seven studies were included in this meta-analysis. The LPA level was obtained and assessed by self-administered questionnaires during follow-up. The diagnostic criteria of MS were in accordance with the new National Cholesterol Education Program’s (NCEP’s) Adult Treatment Program III (ATP III) in the study of Cheriyath *et al*. [13]. The other four studies [12,14,21,22] diagnosed MS according to the original NCEP ATP III. The total sample size of the five articles was 22,023 including 5,084 MS cases. Moreover, the quality evaluation of the included articles is shown in Table 2. All the included literatures were of high quality as they scored 7.

**Table 1:** Characteristics of the five prospective cohort studies

**Included study**	**Region period**	**Follow-up time**	**Ascertainment of LPA level**	**Diagnostic criteria of MS**	**LPA level**	**Age (years) gender**	**Cases/controls**	**Adjusted OR (95% CIs)**	**Adjustment for covariates**
Holme *et al.* (2007) [14]	Norway 1972 to 2000	28 years	Self-administered questionnaires	NCEP ATP III	Sedentary/light	40 to 49 M	337/1,112	1.0	Age, education, triglycerides, smoking, glucose, BMI, treated hypertension and SBP in 1972/1973.
					Moderate		967/3,807	0.98 (0.83 to 1.17)	
					Moderately vigorous		269/1,319	0.83 (0.67 to 1.02)	
					Vigorous		24/141	0.73 (0.44 to 1.22)	
Laaksonen *et al.* (2002) [22]	Finland 1997 to 2001	4 years	Self-administered questionnaires	NCEP ATP III	<270 min/week	42, 48, 54, 60 M	Total:	1.0	Age, BMI, SBP, DBP, antihypertensive medications, glucose, family history of diabetes, triglycerides, insulin and HDL.
					370 to 486 min/week		107/612	0.83 (0.45 to 1.52)	
					≥487 min/week			0.54 (0.28 to 1.04)	
Cheriyath *et al.* (2010) [13]	USA 1987 to 1995	6 years	Self-administered questionnaires	NHLBI and AHA ATP III	Low	45 to 64 M and F	641/2,366	1.00	Age, race, gender, education, smoking, prevalent coronary heart disease, total cholesterol and obesity.
					Middle		975/3,845	0.99 (0.86 to 1.13)	
					Upper		354/1,643	0.90 (0.78 to 1.03)	
Méndez-Hernández *et al*. (2009) [12]	Mexico 2004 to 2006	2 years	Self-administered questionnaires	NCEP ATP III	<30 min/day	20 to 70	Total:	1.00	Age, calories and alcohol intake, smoking, work-place physical activity and education.
					≥30 min/day	M	376/1,484	0.72 (0.57 to 0.95)	
						F	Total:	1.00	
							792/3,634	0.78 (0.64 to 0.94)	
Yang *et al*. (2008) [21]	Finland 1992 to 2001	9 years	Self-administered questionnaires	NCEP ATP III	Inactive	15, 18, 21, 24, 27, 30	Total:	1.00	Age, smoking and education.
					Moderately active		146/961	0.86 (0.58 to 1.29)	
					Active			0.50 (0.29 to 0.86)	
						M	Total:	1.00	
						F	96/1,099	0.79 (0.49 to 1.27)	
								0.20 (0.08 to 0.49)	

AHA, American Heart Association; ATP III, Adult Treatment Program III; BMI, body mass index; CI, confidence interval; DBP, diastolic blood pressure; F, female; LPA, leisure-time physical activity; M, male; MS, metabolic syndrome; NCEP, National Cholesterol Education Program; NHLBI, National Heart, Lung and Blood Institute; OR, odds ratio; SBP, systolic blood pressure.

**Table 2:** Quality assessment of included studies in the meta-analysis

**Included study**	**Representativeness of the exposed cohort**	**Selection of the unexposed cohort**	**Ascertainment of exposure**	**Outcome of interest not present at start of study**	**Control for important factor or additional factor**^**a**^	**Outcome assessment**	**Follow-up long enough for outcomes to occur**	**Adequacy of follow-up of cohorts**	**Total quality score**
Holme *et al.* (2007) [14]	✩	✩	-	✩	✩✩	✩	✩	-	7
Laaksonen *et al.* (2002) [22]	✩	✩	-	✩	✩✩	✩	-	✩	7
Cheriyath *et al.* (2010) [13]	✩	✩	-	✩	✩✩	✩	-	✩	7
Méndez-Hernández *et al*. 2009 [12]	✩	✩	-	✩	✩✩	✩	-	✩	7
Yang *et al*. 2008 [21]	✩	✩	-	✩	✩✩	✩	-	✩	7

A study could be awarded a maximum of one star for each item, except for the item control for important factor or additional factor. ^a^A maximum of two stars could be awarded for this item.

### Meta-analysis

LPAs were divided into three levels (low level LPA, moderate level LPA and high level LPA) in three included studies [21-23]. In the study of Holme *et al*. [14], the moderately and moderately vigorous levels of LPA were considered as moderate level LPA. The study of Méndez-Hernández *et al*. [12] only had low level and moderate level LPA groups. Thus, there were eight sets of data for moderate level LPA versus low level LPA and five sets of data for high level LPA versus low level LPA.

For the moderate level LPA versus low level LPA, the statistical heterogeneity among the studies was not significant (*I*^2^ = 19.9%, *P* = 0.272) (Figure 2), thus the fixed effects model was used. The pooled OR of the moderate level LPA versus low level LPA was 0.89 (95% CI: 0.82 to 0.96, *P* = 0.003). This indicated that the effect of moderate level LPA on reducing the risk of MS was more significant than the low level LPA. For the high level LPA versus low level LPA, the significant heterogeneity (*I*^2^ = 75.0%, *P* = 0.003) (Figure 3) among studies was found and the random effects model was used. The overall OR of the high level LPA versus low level LPA (OR = 0.58, 95% CI: 0.38 to 0.89, *P* = 0.012) demonstrated that high level LPA significantly decreased the risk of MS compared with low level LPA.

**Figure 2:** **Forest plots for the risk of MS associated with the moderate level LPA.** CI, confidence interval; LPA, leisure-time physical activity; MS, metabolic syndrome, OR, odds ratio.

**Figure 3:** **Forest plots for the risk of MS associated with the high level LPA.** CI, confidence interval; LPA, leisure-time physical activity; MS, metabolic syndrome, OR, odds ratio.

### Subgroup analysis

The subgroup analysis by region and gender for the high level LPA versus low level LPA is shown in Table 3. Female (OR = 0.20, 95% CI: 0.08 to 0.49, *P* <0.001) and male (OR = 0.59, 95% CI: 0.43 to 0.82, *P* = 0.002) with high level LPA all have lower risk of MS than with low level LPA. In the subgroup analysis by region, compared with the Europeans with low level LPA, the risk of MS was significantly reduced in Europeans with high level LPA (OR = 0.49, 95% CI: 0.32 to 0.77, *P* = 0.002). There was no significant difference in the risk of MS among the Americans with high level LPA and low level LPA (OR = 0.59, 95% CI: 0.43 to 0.82, *P* = 0.002).

**Table 3:** Forest plots for the risk of MS associated with high level LPA

**Group**	**Number of studies**	**OR (95% CI)**	**Heterogeneity test**		**Significance test (*P*)**
			***P *** **I**^**2**^	**(%)**	
All studies	5	0.58 (0.38 to 0.89)	0.003	75.0	0.012
Area					
Europe	4	0.49 (0.32 to 0.77)	0.112	50.0	0.002
The Americas	1	0.90 (0.78 to 1.03)	-	-	0.137
Gender					
Male	3	0.59 (0.43 to 0.82)	0.578	0.0	0.002
Female	1	0.20 (0.08 to 0.49)	-	-	<0.001
Male and female	1	0.90 (0.78 to 1.03)	-	-	0.137

CI, confidence interval; LPA, leisure-time physical activity; MS, metabolic syndrome; OR, odds ratio.

### Sensitivity analysis

In the sensitivity analysis, no additional studies were found by the application of the trim-and-fill method. For the moderate level LPA versus low level LPA, the pooled OR obtained by the random effects model was 0.88 (95% CI: 0.80 to 0.96, *P* = 0.005). For the high level LPA versus low level LPA, the pooled OR calculated by the fixed effects model was 0.82 (95% CI: 0.72 to 0.93, *P* = 0.002). It indicated that the results of this meta-analysis were not varied in the sensitivity analysis. The stability of the results of this study was confirmed by the sensitivity analysis.

### Publication bias

There was no indication of publication bias based on the Egger’s (*P* = 0.536) and Begg’s test (*P* = 0.196).

## Discussion

MS is highly prevalent in populations around the world. Physical inactivity is one of the major modifiable risk factors for MS [24]. In this meta-analysis, we assessed the association between LPA and the risk of MS. The results indicated that moderate level LPA and high level LPA could decrease the risk of MS. The sensitivity analysis provided evidence for the stability of the results in this study. Consistent results were also obtained in some other published studies. Yu *et al*. reported that PA is associated with a reduced risk of MS among Chinese people [25]. Another article reported that the low levels of childhood PA and aerobic fitness are associated with the presence of MS in adolescents [26]. It suggested that PA needs to begin in childhood to prevent MS.

The subgroup analysis demonstrated that there was no difference in the risk of MS among Americans with high level LPA and low level LPA. The result was different from that in Europeans. The heterogeneity among the studies was weakened in the subgroup analysis. Thus, the difference of region may be one of the sources of heterogeneity. However, the heterogeneity still existed in the subgroup analysis. Further studies need to be undertaken to explore the sources of heterogeneity.

It was reported that regular PA should be performed more frequently (3 to 5 days per week) and for a longer duration (up to 60 minutes) at a lower intensity (approximately 40% to 60% VO_2max_) for metabolic benefits [22,27-29]. PA is a complex and multi-dimensional behavior and affects total energy expenditure which is the sum of the basal metabolic rate [30]. It is well known that PA can reduce fat mass. Even when an exercise program produces no loss in bodyweight, substantial reductions in abdominal subcutaneous and visceral fat can be achieved [31]. Aerobic exercise training also produces favorable changes in plasma lipids and lipoproteins [32]. Miles *et al*. reported that exercise training would alter cholesterol and low-density lipoprotein (LDL) cholesterol when changes in bodyweight and dietary fat reduction are also achieved from the intervention [30]. The study of Hardman *et al*. showed that vasodilation of the arterioles in the exercising muscles would cause a decrease in peripheral resistance [33]. When exercise ceases, cardiac output quickly falls back to pre-exercise levels, but the vasodilation and decrease in peripheral resistance persists for hours [31]. Therefore, it is not surprising in the meta-analysis of 72 trials that endurance training for ≥4 weeks induced significant net reductions of resting and daytime ambulatory blood pressure [34]. In addition, near-daily PA demonstrated positive effects on the immune response [35]. In summary, the association of PA with a reduced risk of MS might relate to energy expenditure, fat mass and blood pressure reduction, and enhance the immune response.

There were some advantages of this meta-analysis. The included studies were all high quality studies and they were all prospective cohort studies. Thus, selection bias and recall bias were avoided to a certain extent. There was no publication bias in the included studies. The results of this meta-analysis were reliable and stable according to the sensitivity analysis.

Some limitations of this study should be discussed. The first limitation was that the articles included were all observational studies. Although we regulated the confounding factors (age, education and smoking) in these studies, the association between LPA and MS would be affected. Further studies are needed to verify the effects of these confounding factors on the results of this study. Second, the PA levels were ascertained by self-administered questionnaires during the follow-up. There were no unified criteria for the level of PA. Thus, the effect of different levels of PA on the risk of MS could not be evaluated. Third, the subjects with high levels of LPA generally had a healthy lifestyle. For them, the intake of dietary fiber, vitamins and other nutrients, which might contribute to maintain metabolic functions and increase the preventive effect against MS, was high. This may affect the investigation of the association between LPA and the risk of MS. Furthermore, the included studies were carried out in Europe and America. It is necessary to develop investigations in Asian countries to assess the versatility of the results in this study.

## Conclusions

In conclusion, moderate and high level LPA significantly decreases the risk of MS. However, more cross-sectional studies with large sample sizes should be carried out to verify this conclusion and further investigate the association between PA and MS by a more scientific approach.

## Abbreviations

ATP III: Adult Treatment Program III; CI: Confidence interval; HDL: High-density lipoprotein; LDL: Low-density lipoprotein; LPA: Leisure-time physical activity; MS: Metabolic syndrome; NCEP: National Cholesterol Education Program; OR: Odds ratio; PA: Physical activity.

## Competing interests

The authors declare that they have no competing interests.

## Authors’ contributions

YH conceived and designed the experiment, and drafted the manuscript. XL acquired and analyzed the data. All authors read and approved the final manuscript.
